The article "Accident Liability Determination of Autonomous Driving Systems Based on Artificial Intelligence Technology and Its Impact on Public Mental Health" was retracted in 2023. Reasons: signs of a paper mill; suspected computer-generated content; unreliable results or conclusions; concerns about the data.

# Accident Liability Determination of Autonomous Driving Systems Based on Artificial Intelligence Technology and Its Impact on Public Mental Health

**DOI:** 10.1155/2022/2671968

**Published:** 2022-08-31

**Authors:** Yineng Xiao, Zhao Liu

**Affiliations:** ^1^Advanced Institute of Information Technology, Peking University, Hangzhou 311200, China; ^2^School of Public Policy and Management, University of Chinese Academy of Sciences, Beijing 100049, China

## Abstract

With the rise of self-driving technology research, the establishment of a scientific and perfect legal restraint and supervision system for self-driving vehicles has been gradually paid attention to. The determination of tort liability subject of traffic accidents of self-driving cars is different from that of ordinary motor vehicle traffic accident tort, which challenges the application of traditional fault liability and product liability. The tort issue of self-driving cars should be discussed by distinguishing two kinds of situations: assisted driving cars and highly automated driving, and typological analysis of each situation is needed. When the car is in the assisted driving mode, the accident occurs due to the quality defect or product damage of the self-driving car, and there is no other fault cause; then, the producer and seller of the car should bear the product liability according to the no-fault principle; if the driver has a subjective fault and fails to exercise a high degree of care; the owner and user of the car should bear the fault liability. This paper analyzes the study of the impact of autonomous driving public on public psychological health, summarizes the key factors affecting the public acceptance of autonomous driving, and dissects its impact on public psychological acceptance. In order to fully study the responsibility determination of autonomous driving system accidents and their impact on public psychological health, this paper proposes an autonomous driving risk prediction model based on artificial intelligence technology, combined with a complex intelligent traffic environment vehicle autonomous driving risk prediction method, to complete the risk target detection. The experimental results in the relevant dataset demonstrate the effectiveness of the proposed method.

## 1. Introduction

Technology changes life; due to the rapid development of intelligent science, human life and work have become faster and more convenient with it. The arrival of the artificial intelligence 5G era and the continuous optimization of roads make the development of self-driving cars more rapid. New things always bring a variety of new problems, self-driving cars are no exception, relevant industry regulations and industrial services should be prepared in advance, and in the context of the rule of the law society, self-driving cars are also subject to the regulation of all aspects of the law. Traffic accidents are the first major safety hazard of motor vehicles. Under the development trend of artificial intelligence, cars are gradually automated to reduce the risk of traffic accidents, and the subjects involved in self-driving cars have also changed, so if they are involved in traffic accidents; the determination of liability subjects in accidents cannot be based entirely on traditional motor vehicle-related legal provisions. This paper discusses the issue of determining the subject of tort liability for traffic accidents involving self-driving cars. The diagram of automatic driving system accident liability determination is shown in Figure 1.

There is a real necessity of studying the issue of determining the subject of liability for traffic accidents of self-driving cars. The first is that the car in the self-driving mode is different from the control subject of ordinary cars in the market [1–3]. The control subject of ordinary cars is the human driver by observing the driving environment to make acceleration, deceleration, and other operating instructions. In traffic accidents that occur in ordinary cars, except for rare car manufacturing defects, operational failures, or road problems, the responsibility for the accident is basically attributed to the human driver who is at fault, and the responsibility for the accident is more direct. Self-driving cars, on the other hand, are not only controlled by humans but also have an autonomous driving system that dominates the car's driving pattern. The self-driving car system designed by technicians can not only drive the car based on the original design but also has the learning ability of artificial intelligence, and there is the possibility of being out of human control. When a self-driving car is involved in a traffic accident, it is unfair to attribute responsibility to the human driver, while the feasibility of attribution is controversial if attributed to the self-driving system. Second, self-driving cars are different from ordinary cars in terms of the subjects involved [4].

In the process of ordinary car operation, generally, only four subjects are involved: car owners, car users, car manufacturers, and car sellers, and the division of labor is relatively simple and clear. In addition to the above-mentioned subjects in the operation of ordinary cars, there are also designers of self-driving systems, software and hardware suppliers, Internet operators, and so on. For example, the designer of the self-driving system must ensure that the design is safe and reasonable; the manufacturer of the car must ensure the quality and safety of the self-driving car; the owner or user of the car must regularly maintain the car to avoid unnecessary safety hazards during the operation of the car. Therefore, in traffic accidents involving self-driving cars, there are many combinations of damage results and causes of action, making it difficult to specify them. Thirdly, there are differences between self-driving cars and traditional motor vehicles in the identification of both the subject of product liability and the subject of tort liability [5–8].

The subject of tort liability in traditional motor vehicle traffic accidents is the actual driver of the motor vehicle or pedestrians on the road, but the driving system of self-driving cars is programmed software, which is only used as a tool and does not have civil rights or capacity to act, but it has the ability to drive intelligently, and these make it difficult to identify the subject of tort liability in traffic accidents involving traditional motor vehicles [9]. As a processed and manufactured product, the damage caused by product defects can be applied to product liability, with the producer and seller of the car bearing the responsibility for damages, but it is different from ordinary products. The determination of product liability requires the user to prove that the product is defective, but because of the high-tech nature of self-driving cars, it is undoubtedly more difficult for consumers to determine that the self-driving system is defective, and the product is dangerous, requiring a great deal of time and some understanding of the profession. In the event of a product defect, consumers may be unable to prove it, making it difficult to determine product liability and the responsibility of the producer of the self-driving car. Based on this, China's current laws and regulations cannot solve the problem of determining the subject of product liability in self-driving car traffic accidents.

The impact of autonomous driving on public mental health is defined from the perspective of psychology, and autonomous driving acceptance refers to the degree to which people express approval or agreement with the situation, process, or conditions of autonomous driving. In studies on public acceptance of autonomous driving, different scholars have elaborated on the meaning of acceptance from a variety of perspectives. To enable comparative analysis among studies, this paper divides public acceptance of autonomous driving into five categories: likelihood and attitude of accepting autonomous driving, level of understanding and trust, perceptions and concerns, willingness to pay, and usage preferences. The likelihood and attitude of accepting autonomous driving refer to the likelihood of accepting autonomous driving and the positive or negative attitudes of different groups in different situations and are usually measured by asking respondents directly whether they are willing to accept autonomous driving or by using an attitude scale. Understanding and trust refer to the public's understanding of and trust in autonomous driving technology and are usually measured by means of scales [10, 11].

In terms of understanding, most studies show that people are not unfamiliar with the concept of autonomous driving and have a certain level of understanding of the functions of autonomous vehicles. Residents who have learned about the features of self-driving but have little experience with riding in them have large differences in their knowledge of self-driving cars from different regions, with residents from South Australia and provincial capitals showing higher acceptance of self-driving relative to residents from other regions. In terms of public trust in self-driving cars, virtual proxy driving similar to that of passengers increases trust in self-driving cars. Perceptions and concerns mainly refer to the benefits people perceive that using autonomous driving can bring, the possible risks, and the technical or social issues that people will actively focus on when discussing autonomous driving [12–14]. The researchers drew conclusions by collecting appropriate information through direct questioning, on the one hand, and by modeling technology acceptance, on the other hand, to investigate the relationship between perceptions and trust/willingness to use. Perceived risk was found to be the main barrier preventing them from using autonomous driving and making the public aware of the benefits that autonomous driving offers is expected to increase acceptance of autonomous driving. From the perspective of concerns, existing research shows that public concerns about autonomous driving include safety, control modes, privacy, and legal liability, with safety being the number one concern in many studies; there are significant differences in the level of safety concerns about autonomous driving among different groups, where older, developed country-dwelling, and female respondents had significantly higher levels of safety concerns about autonomous driving than younger, developing country and male respondents were significantly more concerned about self-driving safety. While fully autonomous vehicles are effective in reducing the number and severity of traffic accidents and responding more sensitively in special emergencies, they also expressed concerns about the ability of autonomous driving systems to handle unexpected situations, legal liability in traffic accidents, and personal privacy.

The main contributions of this paper are as follows. First, it analyzes that with the rapid development of artificial intelligence and information technology, self-driving cars are ushering in a revitalized development in social life. The problems that arise from the identification and assumption of tort liability for damage caused by self-driving cars are increasingly prominent. There are many differences between self-driving cars and traditional cars, so the determination and assumption of tort liability for harm caused by self-driving cars also differ greatly from traditional ones. It is of far-reaching significance to address the determination of liability for accidents caused by self-driving systems and their impact on public mental health, which can promote the efficient resolution of tort disputes caused by self-driving cars, reduce the cost of rights protection, protect the legitimate rights and interests of victims, and maintain social justice, as well as promoting the improvement of the corresponding legal norms and the healthy development of the self-driving car industry. This paper proposes a risk prediction model for autonomous driving based on artificial intelligence technology, combined with a complex intelligent traffic environment vehicle autonomous driving risk prediction method, to complete the analysis of autonomous driving system accident liability determination and its risk to public mental health. The experimental results in the relevant dataset prove the effectiveness of the proposed method.

## 2. Related Work

### 2.1. Autonomous Driving System Accident Liability Determination

The self-driving car is a kind of intelligent robot, which refers to the installation of an artificial intelligence system inside the car, and the installation of a location sensor that senses geographic location outside the vehicle. When the person inside the car enters the destination, the artificial intelligence system automatically decides the driving route according to the relevant program algorithm implanted by the developer in advance and then controls the vehicle by controlling the chassis and steering wheel, replacing the natural human driver in the traditional sense, to realize the position transfer in the body space. Self-driving cars through artificial intelligence, information networks, and other high-tech products and drivers will be liberated to varying degrees, to reduce the probability of motor vehicle traffic accidents, ease traffic congestion, reduce some drivers' driving barriers, and reduce automobile exhaust pollution [15–18]. According to the current international classification standards according to the degree of automation of driverless cars can be divided into L0 to L5 six stages: L0 and L1 stages of self-driving cars and traditional cars are basically close in nature, and driving is mainly completed by the driver; L2 to L4 stages of self-driving cars belong to the “human-machine hybrid driving;” L5 stage will fully realize autonomous driving, and the role of human will dominate the operation of motor vehicles from the driver into a passenger without any driving tasks.

According to the current international standards issued by the American Society of Automotive Engineers, the L0–L4 stages all require varying degrees of driver involvement in the driving process, so the L0–L4 stages of self-driving car damage may be related to the driver's fault. If the accident is caused by the driver's improper operation, the self-driving car as a means of transportation is subject to the same road traffic accident liability as ordinary cars, and the driver, i.e., the user of the self-driving car, is liable for the tort according to the degree of fault. In this paper, we believe that the identification of the tort liability subject, in this case, can be accomplished through the allocation of the burden of proof and the installation of a data recording and monitoring system inside the self-driving car. In case of an accident, the injured party only needs to prove the existence of illegal driving conditions of the self-driving car without the specific improper operation of the driver, while the driver needs to prove that he or she is not negligent in the process of the driving task and has fully exercised his or her duty of care in order to save himself or herself from being liable for the product defects of the self-driving car itself or the runaway accident [19].

The tort liability subject of a self-driving car's product defect is found to be harmful when the self-driving car has a product defect, and the relevant subject shall bear the product tort liability according to the product liability law. Product defects refer to the existence of products that endanger the safety of persons and property other than the product is unreasonably dangerous, including defects in the design, manufacture, storage, and other links. Therefore, in the design, manufacture, sale, and use of different stages, the product designer, product manufacturer, and product seller of self-driving cars are required to exercise due care and attention, and their responsibility is determined according to the extent of their obligations, and then the tort liability subject of self-driving car product defects causing harm is determined. The most essential difference between self-driving cars and traditional cars is that they can learn independently and form experiences to apply according to the algorithms and procedures written by the designer. Through learning, self-driving cars obtain data and information from the surrounding environment, summarize the laws, generate new system rules, and self-adjust according to the rules, resulting in the possibility of their decisions and behavior deviating from the initial procedures and algorithms. It is even more difficult to predict and control the decisions and behaviors that will be made based on the new rules generated by autonomous learning. Because the risk of damage caused by the autonomous driving behavior of self-driving cars is difficult to predict and control, it should not be included in the scope of the designer's, producer's, sellers, or even driver's duty of care and should not be used as the basis for determining the subject of tort liability.

In general, the tort liability of self-driving cars cannot be determined simply by fault liability, strict liability, or vicarious liability but must be determined according to different causes of damage such as driver's fault, product defects, or autonomous driving behavior of self-driving cars. In the field of traditional motor vehicles, Chinese law requires every car owner to purchase compulsory liability insurance for motor vehicle traffic accidents, in addition to a commercial insurance policy. However, in the case of self-driving cars, the self-driving system replaces the driver as the driving subject, and the tort liability of natural persons should be transferred to the self-driving car, and it is obviously unfair if only the car owner purchases insurance [20]. However, the insurance parties, liability limits, and other internal liability mechanisms should be different from the mandatory motor vehicle traffic accident liability insurance. In short, the compulsory liability insurance system can share the risk of damage caused by the autonomous driving behavior of self-driving cars within the society, so that the victims can get timely relief and at the same time can well balance the obligations and responsibilities between the designers, producers, sellers, and drivers and protect the development of the self-driving car industry.

### 2.2. The Impact of Autonomous Driving Systems on Public Mental Health

As an emerging technology, there are still many problems with autonomous driving in terms of laws and regulations, ethics, and other aspects. Therefore, many studies are yet to be conducted on the development of autonomous driving. On the one hand, it is important to fully develop safe and efficient self-driving car technology and continuously improve laws and regulations related to self-driving to promote technological progress and improve the level of traffic intelligence; on the other hand, at the early stage of self-driving car development, we fully investigate the impact of the public's cognitive level and psychological health on self-driving and explore the publics [21, 22]. In addition, from the theoretical aspect, under the current situation that the state strongly supports the research and development of technologies related to self-driving cars and various industries are continuously laying out self-driving, there is very limited research on the Chinese public's perception and acceptance of self-driving cars. Therefore, it is important to explore the public's acceptance and perception of self-driving cars, establish the theoretical basis, and explore the influence of related factors, which is important for the future development direction of self-driving. Second, by comparing the differences in public acceptance and perception of fully self-driving cars and highly self-driving cars, it is an important guideline for the future development direction of autonomous driving.

For self-driving cars, the level of user acceptance determines whether the technology can be used in practice. General acceptance and attitude is the key manifestation of autonomous driving acceptance and application. In contrast to self-driving technology, human definitions of it (e.g., public views, beliefs, attitudes, and acceptance) are a necessary concern for the purchase and payment of the technology; without people buying and using self-driving cars, more investment and production will be futile. As mentioned earlier, there are several scholars who have studied the public's views on self-driving cars in general. There are also studies that have measured the acceptability of self-driving cars in different dimensions [23–25].

The research on the acceptability of self-driving cars was synthesized to construct a model that can explain and predict the acceptability of driverless cars to users. The study addresses different levels and dimensions of driverless car acceptability, including user acceptability, satisfaction needs, attitudes, willingness to use, and actual use. As an emerging technological innovation, self-driving cars have attracted a lot of attention. For a nascent technology, it is common to evaluate the technology by assessing public perceptions, trust, attitudes, and acceptance of the technology. Again, these factors will determine the future direction of self-driving cars, and society is able to shape the technology. Although fully self-driving cars are not yet in human use, it is urgent and necessary to fully understand people's perceptions of them. Foreign research on public perceptions of autonomous driving started early and has a solid research base. Among them, early studies on public perceptions of autonomous driving focused on public opinion, perception, and acceptance, generally using descriptive analysis. They found that the public was attracted to some aspects of autonomous driving, such as safety gains and economic benefits, but had high concerns about the safety, confidentiality, legal liability, and management regulation of autonomous driving.

As autonomous driving has taken off and evolved, research on autonomous driving has emerged, with many studies on public perceptions of autonomous vehicles, and in recent years, more studies have attempted to explore the psychological and socioeconomic factors that determine the public's acceptance of autonomous vehicles and the additional costs they are willing to incur for this technology. Models have also been developed to understand user preferences for vehicles with different levels of automation, as well as preferences for different modes of automated vehicles and their determinants. Regarding public attitudes toward self-driving cars, studies have shown some mixed results. Some studies show that public attitudes toward autonomous driving are positive, while others indicate that respondents show negative attitudes toward self-driving cars.

### 2.3. Autonomous Driving and Artificial Intelligence

As an integrated embodiment of the frontier technologies of the times, such as advanced communication technology, cloud computing technology, and vehicle manufacturing technology, autonomous driving is the future direction of driving technology development and has now been incorporated into the Made in China 2025 plan as an important part of the manufacturing power strategy [26, 27]. Along with the maturity of autonomous driving technology, it can not only assist the driver to complete the driving behavior but also eventually replace the driver to complete the driving independently and solve the driving problems caused by the driver's inexperience, physiological state, personality differences, etc. While fuzzy reasoning can explain and express the process of human choice, an artificial neural network overcomes the subjectivity of fuzzy rules based on the difference in the knowledge base of each person in fuzzy reasoning and completes the inference by objective extraction rules. The fuzzy neural network produced by the complementary advantages of the two can objectively reflect the choice process and give physical meaning to each step, which has a better effect on imitating human behavior, and this approach provides a broader application prospect for autonomous driving [28–30].

Automatic driving technology refers to the use of satellite positioning technology, sensors, cameras, and other devices to collect information about their own environmental conditions and the state of the vehicle and bring the information together to the central processor, through computer technology to analyze and process the vehicle information and calculate the best way to drive the vehicle. Meanwhile, according to the degree of intelligence, automatic driving technology is divided into five levels, and the research object in this paper is fully automatic driving, where the driving right is completely transferred to the driving control system of the vehicle. The driving behavior of the vehicle can be divided into lateral driving behavior, i.e., changing lanes, and longitudinal driving behavior, i.e., driving with the speed. At this stage, the research on the lane changing strategy of autonomous driving is mainly divided into two categories, one is based on real data, with the lane changing prediction accuracy as the goal, to achieve lane changing trajectory control and lane changing decision; the second is to apply the characteristics of autonomous driving in the classical simulation method or driving model and study the driving model suitable for autonomous driving. In the model and simulation for autonomous driving, how to interact and game with the surrounding vehicles through lane change and achieve safe lane change and comfortable lane change are the mainstream research ideas, such as the cooperative lane change of multilane vehicles with the goal of safe spacing between vehicles after lane change, the lane change warning proposed by comprehensive surrounding multivehicle information, and the mixed traffic flow lane change rules considering the impact of automatic truck queues on ordinary vehicles. However, there are few automatic driving lane change rules with the main goal of lane change, higher driving speed, as a consideration, especially on highways where transportation efficiency is pursued.

Neural networks are also known in academic circles as artificial networks or neural-like networks. It is a mathematical model that draws on the structure and function of the biological and human brain and uses computers to process information in the engineering field. Neural networks use the results of modern neuroscience research to simulate the process of data processing by the human brain's activity of remembering and recognizing information. It is a research category of artificial intelligence. Along with the development of science and technology, especially the development of biology, people understand more and more about the brain, and thus neural networks have a broader scope of development. The following recognize some inherent characteristics of neural networks.

Distributed storage of information neural networks stores information in different locations and generally uses many processing units connected to each other to represent specific information, so when the local network is damaged or the input signal is partially distorted, the correct output of the network can still be guaranteed, thus greatly improving the fault tolerance and robustness of the network. Information processing and storage are combined into one neural network. Each processing unit of the neural network has both information processing and storage functions, and the processing units reflect the information memory through the successive intensity changes between them, and the intensity changes and their response to the excitation reflect the information processing function. The ability that parallel coprocessing information neurons can process the received information in parallel is demonstrated by its ability to perform independent operations and processing of information, and the neurons in the same layer can calculate the results simultaneously and pass the output results to the neurons in the next layer. The function of a single processing unit is simple, but the function achieved by a large number of processing units working together is very powerful. The processing of information is self-organizing and self-learning neural networks can improve themselves in the process of continuous learning and can achieve innovation. A neural network can obtain its connection weights and connection structure through learning.

## 3. Methods

### 3.1. Model Architecture

The traditional method for predicting the risk of autonomous vehicle driving cannot extract the characteristic parameters of autonomous vehicle driving behavior, which leads to a large deviation of risk prediction results. Therefore, we propose a complex intelligent traffic environment vehicle autonomous driving risk prediction method. The 3D LIDAR can effectively detect and track the target 360°. The 3D LIDAR is mounted horizontally on the top of the vehicle to ensure that it is on the same level as the vision. The camera and lidar are placed together to avoid the problem of a long target detection process. The target consists of a rectangular frame in a unit space and a collection of obstacle points within the frame. The main purpose of text clustering is to divide the obstacles into several different points, form a collection, and at the same time regulate the collection of points with the help of a rectangular model and then realize the construction of a new target. In the initial three-dimensional point cloud to obtain the initial detection targets, the detection targets will be clustered, while the same type of targets will be divided into a collection; the collection is the target set.

At the same time, the initial point cloud information is collected by sensors and converted into target objects, which effectively simplifies the subsequent processing process and provides convenient targets for analysis, estimates the motion state of the vehicle target, analyzes the driving speed and target behavior, and provides target-level results for planning decisions. The proposed model is shown in Figure 2. (1) *Preprocessing.* Because there is a large gap between 3D LIDAR layers and layers, the farther the distance, the larger the gap will be, and the number of reflected radar points will be reduced accordingly. (2) Connected domain analysis mainly refers to the region consisting of target images with the same pixel values and neighboring pixel values. Among them, connected domain analysis refers to the search of each continuous area in the image, which can represent different connected areas by contours. (3) The minimum envelope area rectangle models the detected target vehicle by the square box model while connecting all the contours of the target to form the minimum rectangular envelope. The minimum envelope area is obtained by rotating the rectangle.

### 3.2. Data Association

Based on this, the complex intelligent traffic environment vehicle target detection also needs to be achieved by data association, through the form of a data association matrix to analyze the target association between the front and back frames, to build the association between the current detection of the acquired target and the previous frame target, and then through the current to drive the already tracked target filter, to update the target motion state. In the following, we mainly use the maximum matching idea of the bipartite graph to optimize the data association matrix into one-to-one matching and obtain the maximum number of matching pairs for the optimized target, in which the optimization of the target is mainly realized by the Hungarian algorithm. The operation flow chart of data association is given in Figure 3.

The detected vehicle targets of each frame are placed into the corresponding target chain table, and the correlation between the two frames before and after the target is analyzed to effectively maintain the motion target chain table and obtain the trajectory of the target vehicle. The trajectory of the motion target is obtained by means of the correlation matrix, in which the data correlation value is calculated as

(1) $$\begin{array}{c} C_{n-\text{ detect}-\text{track}}\left(t\right)=\left[\begin{array}{ccccc} C_{1,1} & C_{1,2}, & \cdots & C_{1,n-\text{track}-1} & C_{1,n-\text{track}}\\ C_{2,1} & C_{2,2} & \cdots & C_{2,n-\text{track}-1} & C_{2,n-\text{track}}\\ C_{n-\text{detect}-1,1} & C_{n-\text{detect}-1,2} & \cdots & C_{n-\text{detect}-1,n-\text{detect}-1} & C_{n-\text{detect}-1,n-\text{track}}\\ C_{n-\text{ detect},1} & C_{n-\text{detec},2} & \cdots & C_{n-\text{detec},n-\text{detect}-1} & C_{n-\text{detec},n-\text{track}} \end{array}\right], \end{array}$$

where *C*_*n*− detect−track_ represents the data correlation value; n-track represents the total number of targets on all tracks; n-detect represents the total number of targets after filtering. The similarity value of the data can be calculated by

(2) $$\begin{array}{c} C_{i,j}\left(t\right)=\frac{1}{\left|x_{t}-{\hat{x}}_{t}\right|+1}+\frac{1}{\left|y_{t}-{\hat{y}}_{t}\right|+1}+\frac{1}{\left|H_{t}-{\hat{H}}_{t}\right|+1}. \end{array}$$

In this equation, ${\hat{x}}_{t}$ and ${\hat{y}}_{t}$ represent the estimated position and vehicle width of the moving target at time *t*. ${\hat{H}}_{t}$ represents the estimated position and vehicle length of the moving target at time *t*−1. *x*_*t*_, *y*_*t*_, and *H*_*t*_ represent the true values of different parameters, respectively; after the calculation of association values, the association matrix is optimized by using the maximum matching and Hungarian algorithms. A one-to-one correspondence is constructed between the currently detected targets and the already tracked targets while abstracting it as a bipartite graph maximum matching problem. *A*_*m*_ is set to represent the set of detected targets; *B*_*n*_ represents the set of tracked targets, the elements in the two sets do not have any connection, there is a one-to-one link, and there can also be a one-to-many link. At the same time, the obtained relationship matrix is converted into a one-to-one correspondence matrix to satisfy the set constraints and finally achieve the target detection.

### 3.3. Feature Parameter Extraction

For the natural driving data attributes and the main factors affecting the risk of automatic vehicle driving, the following parameters are extracted as the feature indicators of vehicle automatic driving classification clustering: the proportion of time when the vehicle driving speed exceeds 80% of the speed limit *η*: vehicle driving speed is an important factor affecting vehicle safety. If the speed is too high, it will reduce the driver's ability to pass curved surfaces or curved paths and also reduce the driver's reaction time to dangerous situations, increasing the probability of accidents. When the speed exceeds 80% of the speed limit, the driver is considered to tend to travel too fast, and the corresponding formula is

(3) $$\begin{array}{c} \eta =\frac{T_{180\%}}{T}\times 100\%, \end{array}$$

where *T* represents the total duration of the vehicle driving on the road; *T*_180%_ represents the total accumulated time of the vehicle driving speed over 80% of the set speed limit value of the road. The average value of vehicle speed $\bar{v}$ and standard deviation *σ*_*v*_: the relevant research results show that there is a close correlation between the average value of vehicle speed and traffic accidents; the higher the value of $\bar{v}$, the greater the probability of traffic accidents. The standard deviation of vehicle speed represents the dispersion of vehicle speed distribution, and the probability of an accident is positively correlated; the following is the detailed calculation formula:

(4) $$\begin{array}{c} \bar{v}=\frac{1}{n}\sum_{m=1}^{n}v_{m},\\ \sigma_{v}=\sqrt{\frac{1}{n}\sum_{m=1}^{n}{\left(v_{m}-\bar{v}\right)}^{2}}, \end{array}$$

where *v*_*m*_ represents the *m*-th speed value of the vehicle in the natural driving process; *n* represents the total number of samples of speed values in the vehicle driving process. The standard deviation of acceleration *σ*_*a*_, the mean value of positive acceleration ${\bar{a}}^{a}$, and the standard deviation of positive acceleration *σ*_*a*^+^_ are calculated as follows:

(5) $$\begin{array}{c} \sigma_{a}=\sqrt{\frac{1}{n}\sum_{m=1}^{n}{\left(a_{m}-\bar{a}\right)}^{2}},\\ {\bar{a}}^{a}=\frac{1}{n}\sum_{m=1}^{n}\left(a_{m}-\bar{a}\right),\\ \sigma_{a^{+}}=\sqrt{\frac{1}{n}\sum_{m=1}^{n}\left(a_{m}^{+}-a^{a+}\right)}, \end{array}$$

where *a*_*m*_ represents the *m*-th acceleration value in the vehicle driving process; ${\bar{a}}^{a}$ represents the overall acceleration value taken in the vehicle driving process; *σ*_*a*^+^_ represents the overall acceleration average value of the vehicle; am + represents the *m* -th positive acceleration value of the vehicle in the driving process.

### 3.4. Risk Prediction

Since it is impossible to accurately obtain information about the surrounding environment and driving behavior of the vehicle during driving in the video, the multisource heterogeneous data involving vehicle collision risk are organized and quantified and reasonably converted into the initial input parameters of the complex intelligent traffic environment vehicle automatic driving risk prediction model. The driving parameters corresponding to vehicle crash risk are quantified and converted into corresponding driving targets by data-driven technology, while a large amount of historical data is selected as the driving source. A part of the data is set as training samples for training and analysis of the subsequently established model; the remaining part is mainly used to test the accuracy of the model prediction results. To fully exploit the quantitative or qualitative information of uncertainty, the data are modeled and analyzed with the help of the confidence rule base inference method. In the confidence rule, the input *X* is used to obtain the weight of the *k*-th rule:

(6) $$\begin{array}{c} w_{k}=\frac{\theta_{k}\prod_{i=1}^{M}\left(\alpha_{i}^{k}\right)}{\sum_{k=1}^{L}\theta_{k}\prod_{i=1}^{M}\left(\alpha_{i}^{k}\right)}, \end{array}$$

where *w*_*k*_ represents the weight value, *α*_*i*_^*k*^ represents the matching degree between the *i*-th input *x*_*i*_ and the reference value *α*_*i*_^*k*^ in the *k*-th rule, *θ*_*k*_ represents the weight value of the *k*-th rule, *M* represents the number of antecedent attributes, and *L* represents the total number of confidence rules. When the calculation of *w*_*k*_ is completed, the posterior confidence structure of the *k*-th specification is discounted and the posterior terms of all the rules are fused using the evidence inference method to obtain the confidence output shown in

(7) $$\begin{array}{c} O\left(X\right)=\left\{D_{j},\beta_{j}\right\}, \end{array}$$

where *D*_*j*_ represents the posterior term, *β*_*j*_ represents the confidence level of *D*_*j*_, and the specific expression is shown in

(8) $$\begin{array}{c} \beta_{j}=\frac{u\left[\prod_{k=1}^{L}\left(w_{k}\beta_{j,k}+1-w_{k}\sum_{i=1}^{N}\beta_{j,k}\right)-\prod_{k=1}^{L}\left(1-w_{k}\sum_{i=1}^{N}\beta_{j,k}\right)\right]}{1-u\left[\prod_{k=1}^{L}\left(1-w_{k}\right)\right]}, \end{array}$$

where *N* represents the total number of posterior terms; *β*_*j*,*k*_ represents the confidence level of the assigned result as *D*_*j*_; *u* represents the range of values of the input variables, which is calculated as follows:

(9) $$\begin{array}{c} u=\left[\sum_{j=1}^{N}\prod_{k=1}^{L}\left(w_{k}\beta_{j,k}+1-w_{k}\sum_{i=1}^{N}\beta_{i,k}\right)-\left(N-1\right)\prod_{k=1}^{L}\left(1-w_{k}\sum_{i=1}^{N}\beta_{i,k}\right)\right], \end{array}$$

where *β*_*j*,*k*_ represents the confidence level of the assignment result *D*_*i*_. The main purpose of the confidence rule base for learning model optimization is to continuously and dynamically adjust the parameter set P so that the optimization objective function can reach the minimum value.

## 4. Experiments and Results

### 4.1. Experiment Setup

In addition to the test methods introduced above, designing reasonable and perfect evaluation schemes and indicators is also a key point when conducting autonomous driving vehicle testing and algorithm evaluation. At present, there is no unified standard for the performance evaluation of autonomous vehicles, and various R&D institutions and research scholars have given evaluation indexes and schemes from different dimensions and focuses. The simulation test evaluation system is shown in Figure 4.

Simulation is a digital virtual testing method consisting of scenarios, vehicle dynamics models, sensor models, algorithms, etc., which allows computer numerical simulation of the system and the whole vehicle of the self-driving vehicle. It uses digital modeling to model the mathematics of the real physical world and validate algorithmic strategies without the need for real-world testing, which has the advantages of high efficiency, low cost, and high freedom partially or fully. Depending on the degree of control of the test object, the simulation can be subdivided into the model in the loop, software in the loop, hardware in the loop, and vehicle in the loop which is further integrated on the basis of HIL. Among them, MIL/SIL is generally used in the software detailed design and unit testing stage to test the single function of the autonomous vehicle; subsequently, HIL testing is used to complete the integration testing of subsystems (including hardware, underlying, and application layer software) and simulate some electrical characteristics; finally, VIL simulation is used to simulate road and traffic environment under laboratory conditions to complete software acceptance and carry out the whole vehicle MIL/SIL/HIL/VIL with the deepening of the integration of test objects, the confidence of test results gradually increases, but the cost also increases accordingly; the comparison of the characteristics of the above different simulation methods is shown in Table 1.

The predicted and real risk levels of each method are compared, and the results of the experiments are shown in Table 2. Analyzing the experimental data in Table 2, we can see that in the process of predicting the risk of automated vehicle driving for 10 different road sections, the prediction results of the proposed method match the real risk level, while comparison methods 1 and 2 have incorrect predictions. The main reason is that the proposed method effectively extracts the characteristics of different vehicle autopilot behaviors in the prediction process, which lays a solid foundation for the subsequent risk prediction, and increases the prediction accuracy of the whole method, which can better grasp the vehicle operation status.

This experiment was written in Python 3.8, using TensorFlow to implement deep learning and using third-party libraries such as TA-lib to calculate technical indicators. The specific configuration is as Table 3.

The training process loss convergence curve and performance improvement are shown in Figures 5 and 6.

### 4.2. Experimental Results

In order to verify the comprehensive effectiveness of the proposed complex intelligent traffic environment vehicle autopilot risk prediction method, the main road of a city was selected as the test site, and the test time was daytime, mainly including cloudy, rainy, and sunny weather conditions. The experiment collected nearly three months of vehicle driving data for experimental analysis, of which the dark curve is the experimental route. Vehicle speed control/(km/h) is in the same road section, using three different methods to predict the vehicle's driving speed, compared with the best driving speed within the road section; the specific experimental results are shown in Figure 7. The analysis of the experimental data in Figure 7 shows that the prediction results of the vehicle driving speed of the research method and the value of the best speed are basically the same, which fully verifies the superiority of the proposed method.

Figure 8 shows the change in the average accuracy of the YOLOv4 algorithm for common road target detection on different data sets before and after the improvement. On the CTS dataset proposed in this paper, the mAP value improves from 85.15% before improvement to 89.91%, an improvement of 4.76%; on the simpler VOC2007 dataset, the detection accuracy can reach a higher level, with the mAP value of 88.90% before YOLOv4 improvement, reaching 91.16% after improvement, an improvement of 2.26%. On the more complex COCO2017 dataset, the detection accuracy did not drop much compared with the CTS dataset, with the mAP value of 81.50% before the improvement of YOLOv4 and 84.16% after the improvement, an improvement of 2.66%, and 88.53%, an improvement of 2.36%. These experimental results show that the improved YOLOv4 algorithm can solve the problems of poor detection of small targets and occluded targets and high miss detection rate so that the algorithm still has a high comprehensive detection ability in complex traffic scenes and is suitable for different traffic scenes and can meet the practical requirements of self-driving cars.

In this section, the improved YOLOv4 algorithm is compared with Faster R–CNN, SSD, YOLO, YOLOv4, and other target detection algorithms on the CTS dataset for experiments, and the selected evaluation metrics are mAP as well as frame rate. The evaluation results of target detection for different algorithms are given in Figures 9 and 10. From the analysis of the evaluation results, the improved YOLOv4 target detection algorithm is far ahead of other algorithms in terms of accuracy rate, reaching 89.91%; in terms of detection speed, the detection speed reaches 35.52 f/s, which is lower than YOLO and YOLOv4, but still meets the real-time requirement of 30 f/s for automatic driving, fully demonstrating the effectiveness of the YOLOv4 improvement algorithm proposed in this paper.

## 5. Conclusion

Self-driving cars follow the trend of artificial intelligence development and have a large economic market and social and cultural influence in the intelligent technology industry. For the legal relationship problems faced in the process of putting this new thing, self-driving cars, into market use, this paper analyzes the determination of the tort liability subjects when self-driving cars are involved in road traffic accidents among them. Since the issue of auto traffic accidents is closely related to the economic interests, personal safety, and rights protection of the people involved in the accident, the determination of the subject of liability is naturally an important part of the resolution of the incident and the protection of human rights. The types of torts that may arise in the event of a traffic accident in the future use of self-driving cars that are identical to and different from those of traditional car accidents have been studied and discussed. The introduction and use of self-driving cars is not only a breakthrough in smart technology but also a challenge to laws and regulations that maintain a stable balance in society. In order to ensure that the accountability of self-driving car traffic accidents in the future can be based on the law, it is imperative to revise the road traffic laws and regulations. This paper investigates the impact of the determination of tort liability subjects and public mental health in self-driving car traffic accidents and proposes a deep learning-based risk detection model for autonomous driving. By revising the relevant laws, we formulate legal norms that are in line with the development of artificial intelligence technology, protect the legal rights and interests of consumers, and ensure the personal and property safety of car users. In the future, we plan to conduct research on the determination of accident liability of autonomous driving systems using graph convolutional neural networks and their impact on public mental health.

## Figures and Tables

**Figure 1:** The diagram of automatic driving system accident liability determination.

**Figure 2:** Model structure.

**Figure 3:** Schematic diagram of data correlation.

**Figure 4:** Simulation test evaluation system.

**Figure 5:** Training process loss convergence curve.

**Figure 6:** Training process performance improvement diagram.

**Figure 7:** Vehicle travel speed prediction results of different methods.

**Figure 8:** Algorithm improvement performance comparison.

**Figure 9:** Comparison of average accuracy of different target detection algorithms.

**Figure 10:** Comparison of frame rates of different target detection algorithms.

**Table 1:** Comparison of simulation test methods.

Simulation method	Model in the loop	Software in the loop	Hardware in the loop	Complete vehicle in the ring
Object under test	Algorithmic models	Target software	Target subsystem	Whole car
Number of test cases	Many	Code	More	Less
Running environment	Design host	Many	Target hardware	Target vehicle
Real-time	Accelerated, real	Design host	Real-time	Real-time
Driver	Time, slow	Accelerated, real	Virtual	Real
Vehicle dynamics	Virtual	Time, slow	Virtual	Real
Sensors	Virtual	Virtual	Virtual or partially	Real
Controllers	Virtual	Virtual	Real	Real
Driving environment	Virtual	Virtual	Virtual or real	Partially real

**Table 2:** Comparison of simulation test methods.

Test road section number	Vehicle autopilot real risk level	Results for predicting the risk of automated vehicle driving		
		Literature of the proposed method	Comparison method 1	Comparison method 2
01	II	II	II	III
02	III	III	III	IV
03	IV	IV	II	IV
04	III	IV	III	IV
05	IV	I	I	I
06	II	II	IV	II
07	III	III	II	I
08	IV	IV	IV	V
09	IV	I	IV	II
10	II	II	II	III

**Table 3:** Experimental environment configuration.

Python	3.8
TensorFlow	2.5.0
Pandas	1.2.4
Numpy	1.19.5
Matplotlib	3.4.2
Scipy	1.6.3
Tushare	1.2.62
TA-lib	0.4.24
Y Finance	0.1.59

## Data Availability

The datasets used during the current study are available from the corresponding author upon reasonable request.
